The article "Effect of Virtual Reality Combined with Intelligent Exercise Rehabilitation Machine on the Nursing Recovery of Lower Limb Motor Function of Patients with Hypertensive Stroke" was published in 2022. Journal: J Healthc Eng.

# Effect of Virtual Reality Combined with Intelligent Exercise Rehabilitation Machine on the Nursing Recovery of Lower Limb Motor Function of Patients with Hypertensive Stroke

**DOI:** 10.1155/2022/2106836

**Published:** 2022-03-03

**Authors:** Xiaoxia Lv, Huan Chen

**Affiliations:** Department of Neurology, Huzhou Central Hospital, Affiliated Central Hospital, Huzhou University, Huzhou 313000, Zhejiang, China

## Abstract

The lower limbs of the human body are stable and flexible weight-bearing joints. They usually perform a variety of complex and subtle jobs whose functions directly affect people's daily lives. The most common type of stroke patients is limb movement dysfunction. 50% to 70% of survivors still have hemiplegic lower limb dysfunction within 2 to 4 years after stroke, which seriously affects their daily life, social participation, functional role, and independence of leisure activities and increases the heavy burden on family and society In order to understand the pathological conditions of ischemic stroke and the role of intelligent sports rehabilitation machines in the diagnosis and treatment of patients with hypertensive stroke, this article collects relevant information through case investigations of patients and interviews with professionals. Using a controlled experiment, the patients were treated in groups, and different treatment plans were used to compare the recovery of the patients' lower extremity movement ability, so as to provide some reference for the subsequent researchers. The results of the study found that stroke patients are more common in the elderly, the incidence rate of the elderly is 6 times that of young adults, and the recurrence rate of hypertensive stroke patients is 10%, which is extremely harmful. The intelligent exercise rehabilitation machine can play a great role in the treatment of patients. It can greatly improve the motor function of the patient's lower limbs. The effect is about 30% higher than that of general treatment methods, and it can also play a certain role in the prognosis of rehabilitation and effectively prevent related postoperative complications. This shows that the intelligent sports rehabilitation machine should raise people's attention in the diagnosis and treatment of patients with hypertensive stroke and increase research and development efforts and promotion efforts, and it can play a greater role in the diagnosis and treatment of patients with hypertensive stroke.

## 1. Introduction

With the overall improvement in the standard of living of Chinese people, the biggest change in people's diet compared to before the reform and opening up is an increase in fat intake, and people's nutritional status is generally good or surplus [1]. The morbidity and mortality of cerebrovascular diseases in my country are showing an increasing trend year by year. Moreover, in recent years, the annual expenditure for cerebrovascular diseases in my country has reached nearly 20 billion yuan, which not only brings a great economic burden to our country but also brings a great physical and mental burden to the families of many patients [2]. Its own characteristics are high morbidity, insufficient attention by people, and rapid progress in treatment that is not timely, resulting in a high disability rate, affecting human life and health and life treatment, and it is one of the main causes of human death [3]. At present, the diagnosis of acute cerebral ischemia is mainly through imaging methods such as computed tomography and magnetic resonance. Clinicians make rapid diagnoses and implement treatment based on clinical experience. The proven effective intervention method for acute cerebral ischemia is vascular recanalization. The key to treatment is to open the blocked blood vessel as soon as possible, save the ischemic penumbra, and avoid serious symptomatic bleeding complications.

The article "Effect of Virtual Reality Combined with Intelligent Exercise Rehabilitation Machine on the Nursing Recovery of Lower Limb Motor Function of Patients with Hypertensive Stroke" was published in 2022. Journal: J Healthc Eng.

When a hypertensive stroke occurs, the blood supply to cerebral blood vessels is blocked due to blood clots causing vascular stenosis and other reasons, resulting in insufficient blood perfusion of brain tissue [4]. In our country, hypertensive stroke accounts for up to 70% of stroke patients. Previous studies have shown that IS can cause a recurrence rate of about 8%–12% in the first year, with an annual recurrence rate of about 3%–8%. Therefore, how to strengthen effectively the secondary prevention effect of IS patients and improve the intensity of secondary prevention is still a problem that needs to be solved urgently. Abnormal lipid metabolism is the main influencing factor of cerebrovascular disease [5]. At present, large sample randomized controlled clinical studies show that intelligent motion recovery machine based on virtual reality to cerebrovascular disease lipid-lowering effect is remarkable, especially in the case of cholesterol lipid-lowering therapy, which can effectively reduce the risk of cardiovascular disease in high-risk patients and can effectively improve the patients with lower limb motor function, thus can be used as a very important method for prevention and treatment of cerebrovascular disease.

For hypertensive stroke, experts at home and abroad also have many studies. Cramer and other scholars found that the functional reorganization of neurons around the injured area, the compensation of the contralateral undamaged motor center, and the activation of the bilateral auxiliary motor area (SMA) can promote the recovery of the damaged motor center. Studies have found that stroke patients undergo repetitive active training in specific situations. After a period of strengthening, the cerebral cortex will undergo a “use-dependent” reorganization phenomenon, which is an activity-dependent functional reorganization [6]. Cheng believes that hypertensive stroke causes extremely serious harm to people. After treatment, more care should be taken to the patients. He provides related psychological care for patients admitted to a hospital for one year to study their effects on the brain. Whether the prognosis of stroke has a positive effect, the results show that after psychological care, the patient's neurological deficit score has increased significantly, indicating that psychological care can play a role in promoting the recovery of patients' neurological function and ability of daily living in patients with hypertensive stroke [7]; In China, research on the treatment of stroke patients started late. Li explored the role of Shuxuening injection in stroke patients. By selecting 60 stroke patients, they were divided into experimental groups and observations. Group, when the patients were treated, the experimental group was injected with Shuxuening injection. The experimental group was given Shuxuening injection during treatment, and the physiological function of the two groups after treatment was recorded. The experimental results found that patients who injected the Shuxuening injection had neurological deficits. It is lower than the observation group, who believes that Shuxuening injection can play a positive role in stroke patients [8]; Tu et al. have made statistics on patients with hypertensive stroke, which is based on the patient's gender, age, incidence, and recurrence. According to the statistical results, the incidence of hypertensive stroke is about 0.58%–0.61%, and the recurrence rate is about 10%–20%. This shows that hypertensive stroke is a threat to people's health. It needs attention [9]. These studies have a certain reference basis for this article, but due to insufficient samples of these studies, too much emphasis on theories, and unreasonable practical programs, there are too many variables in the study, and the conclusions are unconvincing.

The article "Effect of Virtual Reality Combined with Intelligent Exercise Rehabilitation Machine on the Nursing Recovery of Lower Limb Motor Function of Patients with Hypertensive Stroke" was published in 2022. Journal: J Healthc Eng.

This article uses virtual reality technology to realize human–computer interaction. The main innovations are as follows: (1) This topic is based on virtual reality techniques, system modeling techniques, a complete analysis of the characteristics of hardware interactive devices, and the theory of lower limb rehabilitation. The introduction of virtual reality rehabilitation scenes in the lower limb rehabilitation robots have been proposed and designed. (2) The active-assisted control training model of the lower limb rehabilitation robot has been proposed; the selection of hardware modules, plantar pressure collection, and the design of the amplification circuit has been carried out. According to the design criteria of the lower limb rehabilitation control systems, a set of lower limb rehabilitation robot control systems was built. The experimental results are verified, and the control system is stable and responds quickly. (3) The system objectively evaluated the clinical significance of virtual reality combined with intelligent exercise rehabilitation machine in the treatment of hypertensive stroke, explained the harm of hypertensive stroke, and verified the virtual reality combined with intelligent exercise rehabilitation machine in hypertensive stroke The patient's prognosis can play a role in the recovery of exercise capacity. It lightened the burden of rehabilitation medical staff, greatly improved the training effect, and shortened the rehabilitation period.

## 2. Method of Using Virtual Reality Combined with an Intelligent Sports Rehabilitation Machine in Stroke Patients

### 2.1. Virtual Reality Combined with an Intelligent Sports Rehabilitation Machine

Virtual reality technology is an interactive dynamic virtual environment built by sensor technology, computers, and artificial intelligence that can act on human perception to make people feel like they are there [10]. Virtual practice is the product of the rapid development of computers, Internet, information technology, and virtual reality technology. This type of practice is separated from scientific practice and forms a new practice mode. The usual virtual practice refers to the purposeful and two-way object-oriented perceptual activities of the subject in the virtual environment through digital media. Different from traditional practice, virtual practice has the characteristics of real-time interaction, virtual reality, and communication immersion. Its practice process is not restricted by external objective conditions, transcends the limitations of time and space, and can act on objective reality [11–13].

The application of virtual reality and big data will be the general direction of future development, but for the existing medical order rules and the existing information system, it will take more time to realize fully [14]. Virtual reality still has many challenges at the technical and business level, and issues such as capacity and performance issues and security limitations have yet to be resolved.

In the future, the application prospects of the combination of smart medical and blockchain technology are very broad. Important discoveries in the future about smart medicine, artificial intelligence, medical robots, blockchain technology, 3D printing technology, medical data, and biotechnology will be made. These six technological innovations will completely change our traditional medical model. From the perspective of complexity and technical level, the automation of robotic processes is very accurate, and from the perspective of medical accuracy, it is a perfect combination of intelligence [15]. This development process requires the joint efforts of all personnel.

The article "Effect of Virtual Reality Combined with Intelligent Exercise Rehabilitation Machine on the Nursing Recovery of Lower Limb Motor Function of Patients with Hypertensive Stroke" was published in 2022. Journal: J Healthc Eng.

Virtual reality technology is different from traditional media. In a virtual information environment, it is not only a publisher of information but also a dissemination medium and, at the same time, a receiver of information. This kind of media technology itself is a field of information. There is no information center or authority in this field. Every entrance of virtual reality is the receiver, relay, or sender of information. When we are in virtual reality, we may face “dehumanized” virtual objects. This object may be shaped by the subject's consciousness, but it can communicate like a stranger. On the level, we are our own communication, but the object is a materialized ideal object in our own imagination [16]. But unlike the split personality, under the technology of artificial intelligence, the object we conceive can become a dual existence that has both self-awareness and characteristics endowed by the subject. In this communication process, media technology not only creates the subject but also acts as an intermediary and serves as an object receiver. This new trinity of the communication method did not exist before the maturity of virtual reality technology [17]. This article combines virtual reality into the intelligent sports rehabilitation machine, in which the virtual reality technology composition is shown in Figure 1.

Due to many shortcomings and limitations of traditional sports rehabilitation therapy in clinical applications, people propose a more complete rehabilitation training system that can improve the subjective initiative of patients participating in treatment and improve the effectiveness of rehabilitation medicine. Therefore, the intelligent sports rehabilitation machine and virtual reality technology combined application in the field of rehabilitation medicine is the inevitable trend in the development of lower limb rehabilitation training in the future.

### 2.2. Diagnosis and Treatment of Hypertensive Stroke

The treatment of stroke should follow the principles of early detection, early diagnosis, and early diagnosis and treatment. At present, the diagnosis of stroke is mainly through imaging methods such as computed tomography and magnetic resonance. Clinicians make rapid diagnoses and implement treatment based on clinical experience. A proven and effective intervention for stroke is the recanalization of blood vessels. The key to treatment is to open the occluded blood vessels as soon as possible, preserve the ischemic penumbra, and avoid serious complications (symptomatological bleeding) [18]. The current guidelines are based on the time of onset, that is, intravenous recombinant tissue-type plasminogen activator thrombolytic therapy in the hyperacute phase, and certain conditions (blockage of large blood vessels, existence of salvable ischemic brain tissue, no large-scale infarction, within 16 hours of the front cycle, and within 24 hours of the back cycle) are met [19]. The area of brain injury is hypoperfusion for a long time, and it gradually becomes an infarct area. At the same time, the probability of bleeding after thrombolysis will increase. Time is of the essence for patients with acute cerebral ischemia. Only 7%∼13% of patients with acute cerebral ischemia meet the harsh conditions of mechanical thrombus removal. In addition, up to 49% of mechanical thrombectomy patients have poor efficacy. Therefore, intravenous thrombolysis in the hyperacute phase is the main treatment for acute stroke [20].

The article "Effect of Virtual Reality Combined with Intelligent Exercise Rehabilitation Machine on the Nursing Recovery of Lower Limb Motor Function of Patients with Hypertensive Stroke" was published in 2022. Journal: J Healthc Eng.

Modern advanced imaging technology has significantly changed the diagnosis and treatment of stroke. Through neuroimaging technology, such as multimodal imaging technology, the patient's tissue variation, vascular status, and blood perfusion can be quickly obtained, and based on this information, the cause of hypertensive stroke can be quickly diagnosed, and the time window is suitable for thrombolysis. Patients treated for hypertensive stroke can further assist in treatment decisions for hypertensive stroke and improve the benefits of thrombolysis [21]. Personalized diagnosis and treatment of patients is an urgent clinical need today, and one of the most important functions of neuroimaging is to select patients who are suitable for thrombolytic therapy in acute stroke.

CT is the most commonly used and first imaging tool for acute stroke detection. Plain scan CT is relatively sensitive to cerebral hemorrhage, showing high density, with a CT value of up to 90 HU [22]. Early cerebral ischemia showed low density, decreased gray matter–white matter difference, and decreased brain sulci on plain CT. However, the sensitivity to hyperacute cerebral ischemia is low (only 20%–75%), especially for patients with posterior fossa cerebral ischemia. Due to the widespread use of CT equipment and low inspection costs, CT can be used to rule out hemorrhagic stroke quickly. CT of stroke patients is shown in Figure 2.

The article "Effect of Virtual Reality Combined with Intelligent Exercise Rehabilitation Machine on the Nursing Recovery of Lower Limb Motor Function of Patients with Hypertensive Stroke" was published in 2022. Journal: J Healthc Eng.

The incidence of hypertensive stroke is related to the obstruction of blood supply to the blood vessels in the brain. When cerebral hypertension ischemia occurs, the local cerebral blood flow drops sharply, but the brain metabolism continues to continue, which increases the cerebral oxygen uptake rate in the cerebral ischemic area, and the ratio of deoxyhemoglobin to oxyhemoglobin increases [23, 24].

Due to poor blood supply to the brain tissue, postoperative complications are mostly divided into early complications and long-term complications. The former mainly includes incision skin necrosis and incision infection, while the latter mainly includes deformity healing, traumatic inflammation, etc., which have a serious impact on patient's life. Therefore, in the surgical treatment of ischemic stroke, it is necessary not only to make relevant preoperative preparations to select the correct surgical method and surgical approach but also to reduce surgical trauma under the premise of restoring reduction, so as to improve the efficacy of the operation. To reduce the suffering of patients, after treatment, relevant prognostic treatment should also be done to prevent various complications [25].

### 2.3. Diagnosis of Stroke

Due to the complexity of the disease, there are very large inter- and intraindividual differences in its appearance in the image. Diagnosing doctors rely on their own experience to make subjective judgments, and the accuracy of diagnosis is limited by the doctor's experience and knowledge level, and the consistency is poor. With the development of medical imaging technology, the resolution of medical imaging is getting higher and higher, and the image is getting larger and larger [26]. The imaging examination has become the main method of disease diagnosis, and the number of patients is also increasing. The relationship between bioimaging markers and the benefits of thrombolysis is established, and personalized diagnosis and treatment of hypertensive stroke and intelligent thrombolysis is realized, which will help improve the success rate of thrombolysis and reduce the burden on patients. Therefore, it combines the latest artificial intelligence and pattern recognition technology. In terms of technology, computer-aided diagnosis was performed for neuroimaging data of hyperacute hypertensive stroke.

In the implementation process, it is necessary to use an optical model to illustrate how the three-dimensional discrete data field generates, reflects, blocks, and scatters light, so the reasonable selection of the optical model is an important factor in determining the effect of image data rendering [27]. The expression is as follows:

(1) $$\begin{array}{c} \frac{\Delta I}{I}=\frac{\rho *E*\Delta s*\beta }{E}\\ =\rho *\Delta s*\beta . \end{array}$$

When Δ*s* approaches 0,

(2) $$\begin{array}{c} \frac{\text{d}I}{\text{d}s}=-\rho \left(s\right)*\beta *I\left(s\right)\\ =-\kappa \left(s\right)*I\left(s\right). \end{array}$$

As the lighting conditions of the model change, the image will also change with the discovery as follows:

(3) $$\begin{array}{c} I\left(s\right)=I_{0}\exp\left(-\int_{0}^{s}\kappa \left(t\right)\text{d}t\right),\\ t\left(s\right)=\exp\left(-\int_{0}^{s}\kappa \left(t\right)\text{d}t\right). \end{array}$$

From this, we can see that

(4) $$\begin{array}{c} \partial =1-t\left(s\right)=1-\exp\left(-\int_{0}^{s}\kappa \left(t\right)\text{d}t\right). \end{array}$$

When Δ*s* approaches zero, the following differential equation is used to illustrate the change in light intensity:

(5) $$\begin{array}{c} \frac{\text{d}I}{\text{d}s}=T\left(s\right)*\rho \left(s\right)*A\\ =T\left(s\right)*\kappa \left(s\right),\\ I\left(s\right)=I_{0}+\int_{0}^{s}g\left(t\right)\text{d}t. \end{array}$$

For the application of diagnostic imaging in medical treatment, we generally adopt the following formula:

(6) $$\begin{array}{c} x\left(k+1\right)=Ix\left(k\right)+Jv\left(k\right),\;k=1,2,\ldots . \end{array}$$

The quadratic performance indicators are as follows:

(7) $$\begin{array}{c} K=\sum_{k=1}^{\infty }\left[x^{i}\left(k\right)Jx\left(k\right)+r^{i}\left(k\right)cJ\right], \end{array}$$

where the weighting matrix *Q* is

(8) $$\begin{array}{c} Q=\frac{1}{2a^{2}r^{-1}}{\left(\frac{2b^{2}}{a^{2}r^{-1}}p-t\right)}^{-1}\left[a^{2}r^{-1}t^{2}+2\left(1-b^{2}\right)t\right],\\ Q=\frac{1}{2a^{2}r^{-1}}{\left(\frac{2b^{2}}{a^{2}r^{-1}}t-L\right)}^{-1}\left[a^{2}r^{-1}L^{2}+2\left(1-a^{2}\right)L\right]. \end{array}$$

The parameters and the weighting matrix *Q* are brought in to get

(9) $$\begin{array}{c} \left(\frac{2b^{2}}{a^{2}r^{-1}}I_{x}-t\right)Q=\frac{1}{2}t^{2}+\frac{1-b^{2}}{a^{2}r^{-1}}t. \end{array}$$

This is available through the following formula:

(10) $$\begin{array}{c} Q^{2}+\frac{2\left(1+b^{2}\right)}{a^{2}r^{-1}}Q+\frac{{\left(1+b^{2}\right)}^{2}}{{\left(a^{2}r^{-1}\right)}^{2}}I_{x}={\left(Q+t+\frac{1-b^{2}}{a^{2}r^{-1}}I_{x}\right)}^{2}. \end{array}$$

Conventional rehabilitation treatment seldom takes into account the dynamic interaction between the patient and the real-life environment, and due to the limitation of medical resources, it is difficult to provide a variety of therapeutic equipment with functional purposes in actual work. Patients with different types of illness are all trained in the same treatment environment, the environment is less volatile, and one repetitive action can easily disinterest them. Based on the current situation, robot-assisted training has become an emerging treatment method, combined with virtual reality technology to provide specific training situations and develop the best exercise strategy through concentrated and repetitive active training to improve sports functions.

The article "Effect of Virtual Reality Combined with Intelligent Exercise Rehabilitation Machine on the Nursing Recovery of Lower Limb Motor Function of Patients with Hypertensive Stroke" was published in 2022. Journal: J Healthc Eng.

## 3. Nursing Recovery Experiment of Patients' Lower Limb Motor Function

### 3.1. Experimental Analysis Object

Patients with hemiplegia and lower extremity dysfunction who met the inclusion criteria during the recovery period after stroke were selected. The data are mainly obtained from clinical data from the hospitalization department of this state hospital in recent years, as well as statistics from patient field understandings and telephone interviews, which perform classification analysis and are simulated via computer software. A retrospective analysis of the collected data was conducted by collecting clinical data (gender, age at diagnosis or diagnosis, clinical symptoms and signs at the time of admission) of patients with ischemic stroke in a hospital in this province.

### 3.2. Selection Criteria

#### 3.2.1. Inclusion Criteria

1. Meet the 2014 version of the diagnostic criteria for ischemic stroke written by the Cerebrovascular Disease Group of the Neurology Branch of the Chinese Medical Association
2. Patients with right anterior cerebral circulation ischemic stroke confirmed by cranial CT or MRI, aged 45–75 years, disease course 1–6 months, left limb motor dysfunction, and the affected lower limb in Brunnstrom stages III and IV
3. Seat balance ≥ Grade I, with good visual and auditory comprehension and executive ability
4. Good cognitive function (Hasegawa's dementia scale score ≥30 points)
5. The muscle strength of the lower limbs and legs of the affected side is ≥Grade 2 (Lovett grade), and the MAS is ≤Grade II
6. All enrolled patients signed an informed consent form

#### 3.2.2. Exclusion Criteria

1. Poor consciousness, severe cardiopulmonary disease, or other basic diseases that are not suitable for exercise training, such as unhealed fractures, severe pain, and contractures
2. Uncontrolled diabetes, hypertension, and other diseases
3. No voluntary movement of the upper limbs on the affected side
4. Severe anxiety, depression, impaired listening comprehension, command execution ability, poor cognitive function, visual and auditory impairment, and unable to complete the test
5. Family members or patients refuse to participate in the trial

The article "Effect of Virtual Reality Combined with Intelligent Exercise Rehabilitation Machine on the Nursing Recovery of Lower Limb Motor Function of Patients with Hypertensive Stroke" was published in 2022. Journal: J Healthc Eng.

### 3.3. Construction of the Rehabilitation Exercise Machine

The design of the lower limb rehabilitation robot is mainly the building and assembly of the model with the 3D drawing software, ProE. It is mainly composed of a frame, a scene display screen, a handrail, a rocker, a connecting rod, a pedal, a crank, a sprocket, a motor, and a lifter. It is composed of seats, motor sprocket, and other components and uses a gyroscope mouse pad to achieve interactive functions. The virtual model is shown in Figure 3.

### 3.4. Statistics

All data analysis in this article uses SPSS19.0; the statistical test uses a two-sided test; the significance is defined as 0.05; and *p* < 0.05 is considered significant. The statistical results are displayed as mean ± standard deviation (*x* ± SD). When the test data obey the normal distribution, the double T-test is used for comparison within the group, and the independent sample T-test is used for comparison between the groups. If the regular distribution is not sufficient, two independent samples and two related samples will be used for inspection.

## 4. Experimental Analysis of Nursing Recovery of Patients' Lower Limb Motor Function

### 4.1. Lower Limb Function

The purpose of the design of the lower limb rehabilitation training robot is to realize the gradual recovery of patients with lower limb dysfunction to autonomous walking. By controlling the ankle, knee, and hip joints of the lower extremities, the joints of the lower extremities are coordinated to move, and finally, the motion form of the normal lower extremities is simulated. Among them, the walking gait of the human body is an important factor affecting the rehabilitation of the lower extremities. We list the maximum variation range of each joint of the lower limbs of a healthy human body in the three planes and the variation range of each joint of the lower limbs in the three planes when the human body is walking normally, as shown in Tables 1–3.

In summary, the patient uses rehabilitation robots to perform rehabilitation. Under the condition of satisfying the range of human lower limb movement, ellipse trajectory of lower limb movement can be realized, and patients can realize comprehensive rehabilitation of physiology (physiology), psychology, occupation and social life.

Through hospital admission records, we have collected statistics on patients who have received strokes in the hospital and classified them according to the causes of strokes, as shown in Figure 4:

From Figure 4, we can see that the overall number of stroke patients has shown an upward trend year by year. From 2011 to 2020, the overall number of patients has increased by about 50%. Stroke caused by high pressure is an important factor that leads to patients. The proportion of stroke has increased from 24% in 2010 to about 31% in 2020, which requires people's attention. We classify the severity of stroke in patients, as shown in Figure 5.

The article "Effect of Virtual Reality Combined with Intelligent Exercise Rehabilitation Machine on the Nursing Recovery of Lower Limb Motor Function of Patients with Hypertensive Stroke" was published in 2022. Journal: J Healthc Eng.

From Figure 5, we can see that stroke is extremely harmful, and its proportion of patients far exceeds strokes of other causes. It leads to decreased cardiac ejection fraction, decreased cardiac output, and subsequent decreased cerebral blood flow in the patient. In addition, the vascular regulation ability of elderly patients decreases, which further aggravates cerebral blood flow hypoperfusion and causes extremely serious harm to patients.

### 4.2. Changes before and after Treatment

We look at the relevant parameters of patients before and after receiving treatment and compare the changes of patients before and after receiving treatment, so as to understand the treatment effect, as shown in Figure 6:

From Figure 6, we can see that after treatment, the patient's physical skills have improved significantly. Among them, the blood supply and oxygen supply of the patient's brain were significantly improved, and the cholesterol and fat content was significantly improved. After three months of treatment, the treatment effect of the traditional treatment method and the virtual reality intelligent rehabilitation machine is obvious. The virtual reality intelligent rehabilitation machine is significantly better than the traditional treatment effect, and the patient's stroke has been significantly improved.

We classify stroke patients, count the patients' living habits and physical conditions, obtain the cause of the patient's stroke, and then conduct targeted rehabilitation and prognosis so that the patient can recover. The details are shown in Tables 4 and 5.

From Table 5, we can see that bad living habits are an important cause of stroke. Most patients have the habit of smoking and alcohol abuse, which leads to serious hyperlipidemia and high blood pressure, which greatly hinders the patient's health recovery. We compare the rehabilitation prognosis of patients with normal schedules and patients with bad habits, as shown in Figure 7.

Figure 7 shows that poorly scheduled patients have much lower recovery rates and efficiencies than those with normal schedules. This shows that a good lifestyle is very important for the recovery of the patient's prognosis. When rehabilitating stroke patients, we should pay attention to the patient's living habits in order to better recover the patient.

## 5. Conclusion

Studies show that most stroke patients are less aware of the disease and its risk factors and have reduced preventive medication compliance. Therefore, clinicians need to take proactive interventions to raise patient attention and attention to the prevention of stroke recurrence. In particular, it is necessary to clarify the importance and necessity of virtual reality combined with intelligent exercise rehabilitation machine to promote the prevention of stroke in patients and improve their knowledge level. Combining the essential characteristics, technical characteristics, application scope of virtual reality technology, and the theoretical basis of rehabilitation therapy for patients with lower limb motor dysfunction, virtual reality technology is applied to rehabilitation medicine. There are some shortcomings in this article. Due to time and funding constraints, the sample selection of this article is small and does not cover all types of stroke patients. As a result, the experimental results may have some deviations. In future research, the sample should be increased. In future studies, samples and research frameworks should be added. Visualizing remote network virtual scenes is a new direction of rehabilitation medicine. Relying on network technology to realize the remote communication between rehabilitation patients and doctors, this kind of distributed virtual reality technology is also a problem that needs to be solved urgently.

The article "Effect of Virtual Reality Combined with Intelligent Exercise Rehabilitation Machine on the Nursing Recovery of Lower Limb Motor Function of Patients with Hypertensive Stroke" was published in 2022. Journal: J Healthc Eng.

## Figures and Tables

**Figure 1:** Virtual reality technology composition.

**Figure 2:** Patients with stroke.

**Figure 3:** Diagram of the sports rehabilitation organization.

**Figure 4:** The cause of the patient.

**Figure 5:** Proportion of stroke patients: (a) CE: cardiogenic embolism, WI: watershed infarction, HP: hypertension, and UN: unknown cause and (b) HP: hypertension and NO HP: nonhypertension.

**Figure 6:** Before and after treatment for stroke patients.

**Figure 7:** Comparison of patients' prognosis and rehabilitation.

**Table 1:** Range of hip joint changes.

	Parameter name	Spin	Maximum range of motion of joints	Normal walking as the range of motion
Hip joint	Sagittal plane	Buckling	0°–130°	0°–30°
		Straighten	0°–20°	0°–5°
	Coronal plane	Outreach	0°–40°	0°–5°
		Restrained	0°–25°	0°–3°
	Level	External rotation	0°–90°	0°–6°
		Pronation	0°–60°	0°–3°

**Table 2:** Range of knee joint motion.

	Parameter name	Spin	Maximum range of motion of joints	Normal walking as the range of motion
Knee joint	Sagittal plane	Buckling	0°–130°	0°–70°
	Coronal plane	Almost no movement		
	Level	External rotation at 90° of flexion	0°–50°	0°–10°
		Internal rotation at 90° of flexion	0°–25°	0°–6°

**Table 3:** Range of motion of the ankle joint.

	Parameter name	Spin	Maximum range of motion of joints	Normal walking as the range of motion
Ankle joint	Sagittal plane	Dorsal flexion	0°–30°	0°–18°
		Crouching	0°–60°	0°–18°
	Coronal plane	Slight deflection		
	Level			

The article "Effect of Virtual Reality Combined with Intelligent Exercise Rehabilitation Machine on the Nursing Recovery of Lower Limb Motor Function of Patients with Hypertensive Stroke" was published in 2022. Journal: J Healthc Eng.

**Table 4:** Living habits of patients.

Risk factors	Cardiogenic infarction	Noncardiac infarction	Sum	*P* value
Age ≥ 75	35	21	56	0.038
Male	60	18	78	0.052
Smoking	34	9	43	0.032
Drinking	22	7	29	0.014
Hypertension	82	37	119	0.013
Diabetes	32	12	44	0.023
Hyperlipidemia	34	13	47	0.027
Hyperhomocysteinemia	46	24	70	0.095

**Table 5:** Living habits of patients.

Risk factors	OR	95% CI	*P* value
Age ≥ 75	0.935	0.378–1.853	0.038
Male	1.325	0.628–2.987	0.052
Smoking	1.337	0.425–3.286	0.032
Drinking	2.014	0.537–7.638	0.014
Hypertension	0.382	0.172–1.253	0.013
Diabetes	1.079	0.489–2.356	0.023
Hyperlipidemia	3.158	1.289–7.895	0.027
Hyperhomocysteinemia	0.856	0.477–2.235	0.095

## Data Availability

The data that support the findings of this study are available from the corresponding author upon reasonable request.
